The article "Insulin-Like Growth Factor-1 as a Prognostic Marker in Patients with Acute Ischemic Stroke" was retracted in 2022. Reasons: duplicate publication; signs of a paper mill; concerns about the data.

# Insulin-Like Growth Factor-1 as a Prognostic Marker in Patients with Acute Ischemic Stroke

**DOI:** 10.1371/journal.pone.0099186

**Published:** 2014-06-09

**Authors:** Jian-Hua Tang, Li-Li Ma, Tian-Xia Yu, Juan Zheng, Hui-Juan Zhang, Hui Liang, Peng Shao

**Affiliations:** Department of Neurology, Yantaishan Hospital, Yantai, Shandong Province, China; Georgia Regents University, United States of America

## Abstract

**Objective:**

Insulin-like growth factor-1 (IGF-1) has been associated with cardiovascular risk factors and atherosclerosis. The aim of the present study was to evaluate the prognostic value of IGF-1 levels in patients with acute ischemic stroke (AIS).

**Methods:**

All patients with first-ever AIS from August 1, 2012 to August 31, 2013 were recruited to participate in the study. Clinical data were collected. The National Institutes of Health Stroke Scale (NIHSS) score was assessed on admission blinded to serum IGF-1 levels. For the assessment of functional outcome at 90 days Modified Rankin Scale (mRS) was used. On admission, serum IGF-1 levels were determined by chemiluminescence immunoassay. The influence of IGF-1 levels on functional outcome and death was assessed by multivariate logistic regression analysis.

**Results:**

Patients with an unfavorable outcomes and non-survivors had significantly decreased serum IGF-1 levels on admission (P<0.0001 for both). IGF-1 was an independent prognostic marker of functional outcome and death [odds ratio 0.89 (0.84–0.93) and 0.90 (0.84–0.95), respectively, P<0.0001 for both, adjusted for age, NIHSS score and other predictors] in patients with ischemic stroke. Serum IGF-1 levels ≤130 ng/mL was as an value indicator for unfavorable functional outcome (OR 3.31, 95% CI:1.87–5.62; P<0.0001), after adjusting for other significant confounders.

**Conclusions:**

We reported a significant association between low serum IGF-1 levels and unfavorable functional outcome and death.

## Introduction

Stroke is the second most common cause of death and leading cause of adult disability in China [1]. Outcome after ischemic stroke depends on a complex interaction of multiple factors that contribute to the balance towards either a favorable or unfavorable outcome. Biomarkers are attracting increasing attention as potential predictors of outcome in stroke. Rapidly measurable biomarkers to predict illness development, outcome and mortality are pivotal for optimized care and allocation of healthcare resources. A prompt identification of stroke patients at increased risk for adverse outcome interventions could be targeted to those most likely to benefit.

Insulin-like growth factors (IGFs) are peptide hormones that have significant structural homology with insulin. Substantial data suggest that insulin-like growth factor 1 (IGF-1) is a potent cardiomyocyte growth and survival factor [2]. More recently, evidence has accrued to demonstrate that the IGF-1 play an important role in cancer [3], Alzheimer's disease [4], frail [5], oronary atherosclerosis and restenosis [6], ostnatal brain development and in neonatal hypoxia–ischaemia [7], and diabetes associated dementia [8]. Roubenoff et al [9] found that greater levels of IGF-1 are associated with decreased mortality in community-dwelling elderly adults.

The article "Insulin-Like Growth Factor-1 as a Prognostic Marker in Patients with Acute Ischemic Stroke" was retracted in 2022. Reasons: duplicate publication; signs of a paper mill; concerns about the data.

IGF-1 exerts neuroprotective effects in both white and gray matter under different detrimental conditions. It is a key regulator of cell proliferation and an inhibitor of cell apoptosis and necrosis [10]. Several epidemiologic studies have reported an inverse relation between plasma IGF-1 levels and risk of ischemic stroke [11]–[12]. Similarly, Dong et al [13] found that lower IGF-1 levels were significantly related to risk of stroke, independent from other traditional and emerging risk factors in one cohort Chinese patients. Interesting, Selvamani et al [14] found that low-normal levels of IGF-I was associated with increased mortality in ischemic heart disease and stroke. Bondanelli et al [15] also found that circulating IGF-1 might predict functional performance during rehabilitation and ischemic stroke outcome, while another study suggested that high serum IGF-1 levels just after ischemic stroke onset are associated with neurological recovery and a better functional outcome [16]. In fact, because the pathogenesis of stroke was complex and multifactorial, it remains to be established whether the relation is causative. Therefore, the aim of the present study was to evaluate the prognostic value of serum IGF-1 levels in a cohort of Chinese patients with acute ischemic stroke (AIS).

## Subjects and Methods

All patients with first-ever AIS from August 1, 2012 to August 31, 2013 were recruited to participate in the study. The patients were recruited by a single specialized physician (MA LL) according to the World Health Organization criteria. The time from symptom onset to admission should be within 24 hours. Exclusion criteria were intracerebral hemorrhage, malignant tumor, chemotherapy, renal insufficiency (serum creatinine >175 mmol/L), febrile disorders, severe edema, atrial fibrillation, systemic infections and autoimmune diseases. The study also included 100 age-sex matched healthy controls, recruited contemporaneously from the same geographical area. The control subjects had no subjective symptoms of stroke, and had similar exclusion criteria as the patients.

The article "Insulin-Like Growth Factor-1 as a Prognostic Marker in Patients with Acute Ischemic Stroke" was retracted in 2022. Reasons: duplicate publication; signs of a paper mill; concerns about the data.

The demographical data (gender and age) and history of conventional vascular risk factors (diabetes mellitus, hypertension, hyperlipoproteinemia, atrial fibrillation, smoking habit and alcohol abuse) were obtained. Stroke severity was assessed on admission using the National Institutes of Health Stroke Scale (NIHSS) score [17] by a neurologist. Stroke subtype was classified according to TOAST (Trial of Org 10172 in Acute Stroke Treatment) criteria [18]. The clinical stroke syndrome was determined by applying the criteria of the Oxfordshire Community Stroke Project [19]. Brain imaging (either CT or MRI) was performed routinely within 24 hours after admission. MRI with diffusion-weighted imaging (DWI) was available in some patients. In those patients, DWI lesion volumes were calculated by using the formula 0.5×a×b×c (where a is the maximal longitudinal diameter, b is the maximal transverse diameter perpendicular to a and c is the number of 10-mm slices containing infarct) [20]. For the assessment of functional outcome at 90 days, structured interviews were carried out by a trained medical student who was blinded to IGF-1 levels. Functional outcomes were measured with Modified Rankin Scale (mRS). A favorable outcome was defined as a score below 3 on the mRS [21].

This study was approved by the Institutional Review Board of the Yantaishan Hospital, and all participants were informed of the study protocol and their written informed consent was obtained, according to the Declaration of Helsinki.

All blood samples were collected on the first day of admission under fasting state, and IGF-1 was measured in accordance with standard detection methods in the hospital biochemistry department of this hospital. The serum IGF-1 levels were tested by Immulite 2000(Diagnostic Products Corp., Los Angeles, CA) with an analytical sensitivity of 25 ng/mL. In addition, the detection range was 25–1600 ng/mL and the intra and inter assay coefficient of variation <5%. Routine serum biomarkers were also tested by standard detection methods.

Results are expressed as percentages for categorical variables and as medians (interquartile ranges,IQRs) for the continuous variables. The Mann-Whitney U test and Chi-square test were used to compare the two groups. Correlations among laboratory parameters were analyzed using Spearman's rank correlation test. The influence of IGF-1 levels on functional outcome and death was assessed by multivariate logistic regression analysis, after adjusting for the main baseline variables in the univariate analyses(age, the NIHSS score, infarct volume, stroke syndrome, vascular risk factors and other laboratory biomarkers). Results were expressed as adjusted odds ratios (OR) with the corresponding 95% Confidence interval (CI). Receiver operating characteristic (ROC) curves were utilized to evaluate the accuracy of IGF-1 to predict outcome and death. Thereby the area under the receiver operating characteristic curve (AUC) was a summary measure over criteria and cut-point choices. All statistical analysis was performed with SPSS for Windows, version 19.0 (SPSS Inc., Chicago, IL, USA). Statistical significance was defined as p<0.05

The article "Insulin-Like Growth Factor-1 as a Prognostic Marker in Patients with Acute Ischemic Stroke" was retracted in 2022. Reasons: duplicate publication; signs of a paper mill; concerns about the data.

## Results

We studied 168 patients. The median age of patients included in this study was 72 (IQR, 62–83) years and 46.4% were women. The baseline characteristics of the 168 patients were described in Table 1. The median time from stroke onset to inclusion in the study was 4.8(IQR, 3.3–11.5) hours. The median NIHSS score on admission was 7 points (IQR, 3 to 12). An unfavorable functional outcome was found in 55 patients (32.7%) with a median mRS score of 4 (IQR, 3–6). In our study, 25 patients died, thus the mortality rate was 14.9%. Fifty-five patients (32.7%) received thrombolytic therapy with rtPA within the first 3 h of stroke onset.

**Table 1:** Baseline characteristics of acute ischemic stroke patients and control cases.

Characteristics	Patients(n = 168)	Control (n = 100)	p^a^
Age (years), median(IQR)	72(62–83)	72(63–84)	NS
Female sex (%)	46.4	46	NS
The time from symptom to admission (hours), median(IQR)	4.8(3.3–11.5)	—	
Stroke severity at admission, median NIHSS score (IQR)	7(3–12)	—	
Infarct volume(mL, IQR; n = 125)	15(8–28)	—	
Vascular risk factors no. (%)			
Hypertension	72.0	—	
Diabetes mellitus	42.9	—	
Coronary heart disease	32.7	—	
Hypercholesterolemia	41.1	—	
Family history for stroke	23.2	8	0.002
Alcohol abuse	8.9	6	NS
Smoking habit	18.5	13	NS
Clinical findings median(IQR)			
BMI (kg m^−2^)	25.3(21.8–28.4)	23.9(21.8–26.3)	0.012
Heart rate (beats min^−1^)	81(70–94)	79(69–90)	NS
Temperature (°C)	36.9(36.5–37.4)	36.5(36.2–36.8)	NS
Systolic blood pressure(mmHg)	159(142–173)	128(105–134)	<0.0001
Diastolic blood pressure(mmHg)	94(81–101)	82(74–87)	0.003
Stroke etiology no. (%)		—	
Small-vessel occlusive	23.2		
Large-vessel occlusive	21.4		
Cardioembolic	31.0		
Other	12.5		
Unknown	11.9		
Stroke syndrome no. (%)		—	
TACS	18.5		
PACS	38.1		
LACS	19.0		
POCS	24.4		
Laboratory findings (median, IQR)			
Leucocyte count (×10^3^ m L^−1^)	8.6(7.2–10.1)	8.2(6.8–8.9)	0.042
Glucose(mmol L^−1^)	6.59(5.51–7.49)	5.48(5.02–5.99)	0.002
Hs-CRP(mg dL^−1^)	0.66(0.31–1.03)	0.25(0.12–0.36)	<0.0001
HCY(umol L^−1^)	18.9(13.4–25.7)	12.8(10.2–15.3)	0.006
D-dimer(mg L^−1^)	0.95(0.45–2.45)	0.30(0.15–0.69)	<0.0001
IGF-1(ng mL^−1^)	127(106–156)	155(138–176)	<0.0001

IQR, interquartile range; TACS, total anterior circulation syndrome; LACS, lacunar syndrome; PACS, partial anterior circulation syndrome; POCS, posterior circulation syndrome; NIHSS, National Institutes of Health Stroke Scale; Hs-CRP, High-sensitivity -C-reactive protein; NS, not significant.

a *p* value was assessed using Mann-Whitney *U* test or χ2 test.

The article "Insulin-Like Growth Factor-1 as a Prognostic Marker in Patients with Acute Ischemic Stroke" was retracted in 2022. Reasons: duplicate publication; signs of a paper mill; concerns about the data.

The median serum IGF-1 levels were significantly (P<0.0001) lower in AIS as compared to control normal cases (127; IQR, 106–156 ng/mL and 155; IQR, 138–176 ng/mL, respectively; Figure 1.). There were inverse correlation that linked the levels of IGF-1 to the NIHSS (r = −0.422, P<0.0001; Figure 2a.) and Hs-CRP levels (r = −0.162, P = 0.036; Figure 2b). There was modest correlation that linked the serum IGF-1 levels to age(r = −0.235, P = 0.002). See the Figure S1. There was no significant difference serum IGF-1 levels between men and women (130; IQR, 103–158 ng/mL and 126; IQR, 112–155 ng/mL, respectively; P = 0.745).

**Figure 1:** Serum IGF-1 levels in acute ischemic stroke patients and control group. Mann–Whitney U-test. All data are medians and in-terquartile ranges (IQR). Significantly higher in stroke patients as compared to control cases (P<0.0001).

**Figure 2:** Correlation between serum IGF-1 levels and others predictors. (a) Correlation between the serum IGF-1 levels and the National Institutes of Health Stroke Scale (NIHSS) score; (b) Correlation between serum IGF-1 levels and Hs-CRP;(c) Correlation between serum IGF-1 levels and infract volume;(d) Correlation between serum IGF-1 levels and HCY.

In this study, 125 patients' MRI data were available, there was a negative correlation between serum levels of IGF-1 and the infarct volume (r = −0.258, P = 0.0001; Figure 2c.). In addition, there were no significantly correction between serum levels of IGF-1 and others variables, namely, stroke etiology, stroke syndrome, glucose and HCY (P>0.05). See the figure 2d.

Serum IGF-1 levels in patients with an unfavorable outcome were significantly lower than those in patients with a favorable outcome (114[IQR, 95–124] vs 146 [IQR, 122–165] ng/mL; p<0.0001; see the figure 3a). In univariate logistic regression analysis, we calculated the ORs of log-transformed IGF-1 levels as compared with the NIHSS score, infarct volume and other risk factors. With an unadjusted OR of 0.84(95% CI, 0.76–0.89; P<0.0001), IGF-1 had a strong association with unfavorable functional outcome. After adjusting for all other significant outcome predictors, IGF-1 remained can be seen as an independent unfavorable outcome predictor with an adjusted OR of 0.89 (95% CI, 0.84–0.93; P<0.0001). See the table 2.

**Figure 3:** Serum IGF-1 levels in different groups. (a) Serum levels of Lp(a) in patients with favorable outcomes and unfavorable outcomes; (b) Serum levels of Lp(a) in survivor and non- survivor.

The article "Insulin-Like Growth Factor-1 as a Prognostic Marker in Patients with Acute Ischemic Stroke" was retracted in 2022. Reasons: duplicate publication; signs of a paper mill; concerns about the data.

**Table 2:** Univariate and multivariate logistic regression analysis for outcome and mortality.

Parameter	Univariate Analysis			Multivariate Analysis		
	OR a	95% CI a	*P*	OR a	95% CI a	*P*
Predictor: functional outcome						
IGF-1 (increase per unit)	0.84	0.76–0.89	<0.0001	0.89	0.84–0.93	<0.0001
Age (increase per unit)	1.06	1.03–1.09	<0.001	1.06	1.04–1.08	<0.001
Glucose (increase per unit)	1.08	0.99–1.21	0.015	1.06	0.98–1.22	0.023
Hs-CRP (increase per unit)	1.06	0.97–1.15	0.004	1.05	0.96–1.22	0.009
Infarct volume(increase per unit)	1.19	1.07–1.28	0.002	1.12	1.01–1.22	0.006
NIHSS (increase per unit)	1.16	1.08–1.26	<0.0001	1.14	1.03–1.19	<0.0001
Predictor: death						
IGF-1 (increase per unit)	0.86	0.80–0.90	<0.0001	0.90	0.84–0.95	0.006
Age (increase per unit)	1.08	1.02–1.16	<0.001	1.07	1.03–1.10	<0.0001
Glucose (increase per unit)	1.03	1.00–1.08	0.001	1.02	0.99–1.08	0.002
Hs-CRP (increase per unit)	1.11	1.04–1.19	<0.001	1.09	0.99–1.27	0.003
Infarct volume(increase per unit)	1.22	1.10–1.30	0.005	1.15	1.07–1.26	0.009
NIHSS (increase per unit)	1.18	1.10–1.30	<0.0001	1.16	1.08–1.20	<0.0001

a Note that the odds ratio corresponds to a unit increase in the explanatory variable.

OR, odds ratio; CI, confidence interval; Hs-CRP, High-sensitivity -C-reactive protein; NIHSS, National Institutes of Health Stroke Scale.

Base on ROC curve, the optimal cutoff value of serum IGF-1 levels as an indicator for unfavorable functional outcome was projected to be 130 ng/mL, which yielded a sensitivity of 84.5% and a specificity of 82.4%, with the area under the curve at 0.885 (95%CI, 0.778–0.936). In multivariate analysis, serum IGF-1 levels ≤130 ng/mL was as an value indicator for unfavorable functional outcome (OR 3.31, 95% CI:1.87–5.62; P<0.0001), after adjusting for other significant confounders.

Serum IGF-1 levels in 25 patients who died were significantly lower as compared with patients who survived (96[IQR, 89–121] vs 132[IQR, 115–166] ng/mL, respectively, P<0.001; see the figure 3b). After adjusting for all other significant predictors, IGF-1 level remained an independent predictor for mortality with an OR of 0.90 (95% CI, 0.84–0.95; P = 0.006). See the table 2.

## Discussion

In this study, we found that serum IGF-1 levels were significantly reduced in cases of first AIS compared to control cases. When adjusting for other possible risk factors, reduced IGF-1 levels were independent predictor for unfavorable functional outcome and mortality, and serum IGF-1 levels ≤130 ng/mL were associated with an 3.31-fold increase in AIS patients with unfavorable functional outcome. Furthermore, we found that the serum IGF-1 levels dropped with increasing severity of stroke as defined by the NIHSS score, and there was an inverse correlation that linked the levels of IGF-1 to the infarct volume.

The article "Insulin-Like Growth Factor-1 as a Prognostic Marker in Patients with Acute Ischemic Stroke" was retracted in 2022. Reasons: duplicate publication; signs of a paper mill; concerns about the data.

Our conclusion was consistent with several pervious studies. Bondanelli et al [15] suggested that circulating IGF-1 may predict functional performance during rehabilitation and ischemic stroke outcome, while another study found that serum IGF-1 levels correlate to improvement of functional outcome after ischemic stroke [22]. Similarly, De Smedt et al [16] reported that high serum IGF-1 levels just after ischemic stroke onset are associated with neurological recovery and a better functional outcome. Interestingly, Åberg et al [23] found that variation in rs7136446 of the IGF-1 gene associates with post-stroke outcome in relatively young IS patients in a Scandinavian population. In the present study, no difference in IGF-1 levels was observed between genders. Many other studies also failed to demonstrate distinction between genders [24]–[25]. Previous studies indicated that systemic administration of IGF-1 injection results in a decreased infarct volume [26]-[27]. We also found an inverse correlation that linked the levels of IGF-1 to the infarct volume.

Low level of IGF-1 may ***play a role in the process of AIS progression***. First, impaired insulin/IGF-1 signaling had already been linked to increased oxidative stress and mitochondrial dysfunction in neuronal cells [4]. Hong et al [28] hypothesize that IGF-1 may affect tau phosphorylation through the inhibition of glycogen-synthase kinase-3 in neurons. ***Second***, IGF-1 can regulate cell cycle progression and mitogenesis. IGFs may also function as survival factors by decreasing apoptosis in various cells. Third, among the various growth factors involved in atherosclerotic plaque development, IGFs play a relevant role. Type I IGF receptors are present on smooth muscle cells [29], inflammatory cells [30], and arterial endothelial cells [31] within the atherosclerotic lesion. Macrophage accumulation is an early event in atherosclerosis. It is likely that macrophage-derived IGF enhances cellular LDL uptake and degradation and also the macrophage cholesterol esterification rate [30]. Fourth, IGFs also serve beneficial effects at the vessel wall after injury. It is reasonable to assume that local IGF-1 production may play a role in regenerating the elastic layer. Lastly, Sohrabji et al [32] found that oestrogen-mediated neuroprotection is critically dependent on IGF-1 signaling, and specifically focus on microglia as the source of IGF-1 and the locus of oestrogen–IGF-1 interactions in stroke neuroprotection.

The article "Insulin-Like Growth Factor-1 as a Prognostic Marker in Patients with Acute Ischemic Stroke" was retracted in 2022. Reasons: duplicate publication; signs of a paper mill; concerns about the data.

Some limitations of this study should be consideration. First, long term follow-up data are lacking. Further studies are needed to determine whether serum IGF-1 levels predicts long term outcomes after a stroke in our population. Second, serum IGF-1 levels were only measured once at admission, this study yielded no data regarding when and how long IGF-1 is elevated in these patients. Thus, additional measurements in the days after would have been of interest. Furthermore, biological effects and bioavailability of IGF-1 are modulated through IGFBPs, which control IGF-1 access to cell surface receptors. Unfortunately, we did not have IGFBPs available, and therefore our results do not fully represent biologically active IGF-1. Finally, data derived from a single-centre study always need to be replicated in larger multicentre studies.

## Conclusions

Our study suggests that reduced serum IGF-1 levels are a useful tool to predict unfavorable functional outcome and mortality 90-day after AIS and have a potential to assist clinicians.

## Supporting Information

Figure S1 Correlation between serum IGF-1 levels and age. (a) Correlation between the serum IGF-1 levels and age in the patients with stroke; (b) Correlation between the serum IGF-1 levels and age in the men patients; (c) Correlation between the serum IGF-1 levels and age in the women patients.
(TIF)
